RETRACTED

# Evaluation of Knowledge, Attitude, and Practice of Health Practitioners towards Fertility Preservation in Cancer Patients in an Environmental Region of Saudi Arabia

**DOI:** 10.1155/2022/6404837

**Published:** 2022-06-06

**Authors:** Ramya Ahmad Sindi, Marwah Salem Bagabas, Leen Mamdoh Al-Manabre, Raghad Zahi Al-Sofee, Raneem Yousef Rednah, Shrooq Meshal Al-Jahdali

**Affiliations:** Laboratory Medicine Department, Umm Al-Qura University, Makkah, Saudi Arabia

## Abstract

**Background:**

Cancer patients face multiple challenges, such as infertility caused by exposure to gonadotoxic agents and gonadal irradiation during cancer treatment. Little is known about the health practitioners' knowledge and practice regarding fertility preservation and its available options in Saudi Arabia. Thus, this study is designed to evaluate the level of knowledge, attitude, and practice (KAP) towards fertility preservation in cancer patients among health practitioners in an environmental region in Saudi Arabia.

**Methods:**

The cross-sectional study was carried out between September 2020 and January 2021. A self-administered questionnaire was distributed among health practitioners from a variety of specialties who work closely with cancer patients.

**Results:**

Out of 100 participants, 90% need more knowledge about fertility preservation. The lack of fertility preservation clinics in the patient's area and its unaffordable expenses significantly influenced the health practitioners' attitude towards fertility preservation discussion with cancer patients. The results revealed that 92% of the participants agreed that the Saudi Ministry of Health should establish practice guidelines and provide fertility preservation services for cancer patients.

**Conclusions:**

The present study showed that clinical practitioners' knowledge remains insufficient. Education of health practitioners and the establishment of practice guidelines and fertility preservation clinics for cancer patients are required.

## 1. Background

Cancer is the second-highest cause of death globally, resulting in millions of deaths all over the world. According to the Global Cancer Observatory (GCO), a platform that follows The World Health Organization (WHO), approximately about 19 million new cancer cases worldwide were recorded in 2020, with 9.9 million deaths across both genders [1]. In Saudi Arabia, 27,885 patients were diagnosed, and 13,069 deaths were reported from both genders in 2020. Among females, the most common types of cancer were breast cancer, followed by thyroid cancer and colorectal cancer. In contrast, among male patients, colorectal cancer was the most prevalent, followed by Non-Hodgkin lymphoma (NHL) and leukemia [2].

RETRACTED

Cancer patient faces multiple challenges, along with being diagnosed with cancer. In the past, the main priority for cancer patients was to survive cancer despite any other complications. However, the focus now has changed from treating cancer alone to providing treatment and avoiding long-term consequences, which resulted from cancer therapy such as infertility [3]. According to The World Health Organization (WHO), infertility is defined as the inability or failure to establish pregnancy after one year of trying with regular unprotected sexual intercourse [4]. Infertility rises among cancer survivors, and it is usually associated with significant social, psychological, and economical effects. Preserving cancer patients' fertility before being treated for cancer is highly recommended [5].

The American Society of Clinical Oncology (ASCO) recommended that the possibility of infertility and fertility preservation options must be discussed with a cancer patient. In addition, a cancer patient should be referred to a fertility preservation clinic for consultation before cancer treatment [6, 7]. Despite these fertility preservations guidelines and regulations, a large number of previous studies reported that some health practitioners including oncologists are lacking awareness regarding fertility preservation options before cancer treatments. Therefore, the number of patients' referrals to fertility preservation clinics remains low [8–10].

In Saudi Arabia, the patient bill of Rights and Responsibilities by the Saudi Ministry of Health (MOH) righted that the patient must be informed regarding the possibility of infertility due to cancer and its negative effects and referred to an infertility consultant before undergoing cancer therapy [11–13]. However, fertility preservation of cancer patients is still a challenging issue, and the practice of referral and consulting is not yet fully adapted among Saudi health practitioners.

### 1.1. Cancer Therapy and its Impacts on Fertility

Cancer and its further treatments may induce negative impacts on an individual's fertility. This includes fatigue, loss of sexual desire, and temporal or permanent infertility [5]. These effects are mainly depending on the cancer type, stage, and site. In addition, it depends on the provided type of cancer therapy as the following:

#### 1.1.1. Chemotherapy

It is a group of cytotoxic drugs which are used to shrink the tumor before surgery or terminate the cancer cells. However, it has considerable side effects on the fertility of both males and females [14–16]. Chemotherapy treatment can either reduce fertility or lead to infertility. Its impacts depend on several factors, including the type of cancer and stage, dose and duration, and patient's age. In females, the number of primordial follicles is fixed since birth [17, 18]. The chemotherapy breaks down the DNA strands, increases apoptosis, and decreases stromal function [13]. This leads to changes or stopping of the menstrual cycle temporarily. However, this effect is revised after stopping cancer treatment. Although returning normally to the menstrual cycle does not mean returning to fertility since the ovarian reserve could be low or diminished. Treating cancer by chemotherapy could also stop the menstrual cycle permanently, leading to infertility in some cases [13].

RETRACTED

Whereas in males, chemotherapy reduces testosterone levels, affecting sexual functions [19]. Moreover, it damages the spermatogenesis process, which reduces the number of sperms leading to azoospermia [20, 21]. Azoospermia is a medical condition in which the patient has no sperm in his ejaculate. There are two types of Azoospermia: non-obstructive and obstructive azoospermia. The former refers to the absence of sperm in the ejaculate due to the failure of sperm production, whereas the latter refers to the absence of spermatozoa in the ejaculate despite normal spermatogenesis [22, 23].

#### 1.1.2. Radiotherapy

Another widely adopted option for treating cancer, radiotherapy is where an ionized radiation beam is used to reduce the number of cancer cells and destroy it by damaging their DNA [24, 25]. Radiotherapy has a significant effect on fertility, and this mainly depends on several factors including the site of radiation, the age of the patient, and the dose of treatment. In the case of ovarian cancer, it has been shown that pelvic irradiation could cause a loss of elasticity of the uterus and blood vessels in the endometrium, which leads to miscarriage and pregnancy loss [12]. Moreover, the age of the patient plays a role in the impact of the radiation. A previous study has demonstrated that young patients showed fewer side effects on their fertility and a higher recovery rate than older patients [14]. Furthermore, high doses of pelvic irradiation may greatly damage the sperm and oocytes [13]. In females, when radiation therapy is focused on the pelvic region, it affects the ovaries by destroying the ovarian follicles' DNA, which, therefore, decreases the ovarian follicular number and affects the hormone production. This leads to failure of the uterine function and early stages of menopause. Uterine dysfunction may also be associated with the reduction in uterus size and endometrium damage.

In males, cancer radiotherapy affects the testes and epididymis. It has been demonstrated that pelvic irradiation decreases sperm motility and count by impairing sperm production and increasing the rate of mortality and apoptosis. In addition, radiotherapy may induce a mutagenic effect by increasing sperm DNA abnormalities. Consequently, lower fertilization rate, hypo-fertility, or infertility may occur [26, 27].

RETRACTED

#### 1.1.3. Surgical Treatment

Surgical treatment is widely used to treat uterine cancer and ovarian cancer in females and testicular cancer in males [13]. In cases of ovarian cancer, ovaries removal leads to changes in the vagina and early menopause. As a result, this will impact women's confidence and influence their psychological state [5].

In cases of testicular cancer, orchidectomy or testicles removal from one or both testes decrease the sperm concentration by 50% in comparison to a normal individual [28]. In the case of cystectomy or prostatectomy, it has been shown that patients may suffer from severe azoospermia and erectile dysfunction [29].

### 1.2. Fertility Preservation

Fertility preservation is usually defined as a process of preserving reproductive cells including oocytes, sperm, and embryos, or reproductive tissues including ovarian and testicular tissues to enable individuals to start a family at a time of their choice when their fertility is compromised [30]. The main objective of fertility preservation intervention is to minimize the primary disease burden and more importantly to ensure maintaining or preserving the reproductive health [31].

Oncofertility is a common term for fertility preservation in cancer patients. For individuals who are diagnosed with cancer, fertility preservation is a significant thought when there is a chance that cancer treatment may influence their fertility. Fortunately, there are currently tremendous fertility preservation options that are accessible to cancer patients, and there are numerous individuals who have had the option to begin a family after cancer treatment [32].

With regard to fertility preservation in Saudi Arabia, the Islamic Fatwas were in good agreement with the Saudi System of Fertilization and Embryology Units. In 21-11-1424 H, the system declares that the intervention of third-party reproduction such as sperm, oocytes, and embryo donor/banking is prohibited by law and religion. In addition, it states that fertility preservation options such as embryo freezing can only be offered to married couples, and in case of divorce or death, the frozen embryos must be destroyed [33].

### 1.3. Fertility Preservation Options for Women

#### 1.3.1. Cryopreservation

It is a process used to safely preserve human tissues using liquid nitrogen vapor at shallow temperatures at −196°C. Such a technique is important to stop cell degradation and aging by reversibly halting the metabolism. Furthermore, it maintains the tissue's structure and preserves the tissue's ability to develop and grow after freezing [34]. Cryopreservation has numerous methods, including slow freezing, conventional vitrification, and ultrarapid vitrification [35].

- Oocytes Cryopreservation
- It is a common approach to preserving fertility for postpubertal single girls [36]. The ovaries are stimulated then; mature oocytes are extracted, frozen, and stored for future use. The frozen oocytes can be used in IVF/ICSI techniques [13].
- Ovarian Tissues Cryopreservation
- A surgical procedure for prepubertal and postpubertal [27]. The ovarian tissue is extracted surgically, then fixed in a liquid preservative, cut into thin slices/pieces, and carefully soaked and stored for future use [28]. The ovarian tissue can be transplanted back into the body following cancer therapy to restore ovarian function [14].
- Embryo Cryopreservation
- It is an option offered for women before undergoing cancer therapy. This procedure involves ovarian stimulation to produce multiple oocytes. Two to three weeks after, mature oocytes are retrieved, and in vitro fertilized. The resulted viable embryos are chosen to be frozen and then stored for future use [27].

RETRACTED

### 1.4. Fertility Preservation Options for Men

#### 1.4.1. Sperm Extraction

It is a method to preserve fertility in men and postpubertal boys with azoospermia [27]. This procedure is performed before starting cancer treatment with chemotherapy or radiotherapy [29]. It includes passing a tiny needle into the epididymis or the testes surgically to collect the sperm cells, which will be frozen by one of the cryopreservation methods [14]. Extracted sperm are stored for future use in the assisted reproduction technologies (ART) including In Vitro Fertilization (IVF), Intrauterine Insemination (IUI), and Intracytoplasmic Sperm Injection (ICSI) [29].

#### 1.4.2. Radiation Shielding

A technique used for patients who are treated with radiotherapy, where special shields are placed over the testicles during radiation to reduce the negative effects of radiation. Nevertheless, it does not protect against chemotherapy or total body irradiation [14]. There are several types of shields, such as the calm lead shield [30].

#### 1.4.3. Testicular Transposition

A surgical method is used for prepubertal boys to protect their fertility against radiation. During this procedure, the testis is transposed from the irradiation site, then wrapped in silicon, and placed in the abdomen's anterior wall before starting the therapy to minimize the radiation effects. Following cancer recovery, testis can be surgically transferred to its position and fertility is restored within a year to two years [30].

RETRACTED

### 1.5. Aim of the Study

The current study aims to evaluate the level of knowledge, attitude, and practice towards fertility preservation in cancer patients among health practitioners in an environmental region of Saudi Arabia.

## 2. Methods

This cross-sectional study was conducted to evaluate the level of knowledge about attitude and practice towards fertility preservation in cancer patients among health practitioners who work closely with cancer patients in the Makkah region. The study was conducted between September 2020 and January 2021. Ethical approval (AMSEC 27/1-3-2020) for the study was obtained from the Institutional Ethics Committee at Umm Al-Qura University. The instrument of the study was a self-administered closed-ended questionnaire with a brief introduction to explain the objectives of the survey. The study's questionnaires were randomly distributed to any health practitioners who work closely with cancer patients, and the study participants included 100 health practitioners from a variety of specialties such as medical and clinical oncologists, surgeons, hematologists, nurses, and laboratory specialists, anesthesiologists, pharmacists, and radiologists. In addition, the study participants were asked to sign the written informed consent form to maintain the privacy of their information and were informed that their participation is voluntary and that they can withdraw from the questionnaire at any time.

The current questionnaire was designed and developed by the authors of this study using the Google Forms tool. It was provided in the English language only. The link to the questionnaire was generated and sent as a WhatsApp message to the participated health practitioners' phone numbers or as a Twitter message on their personal Twitter social media accounts. The questionnaire consisted of 18 closed-ended questions which were divided into four main sections. These include the knowledge, attitude, and practice of health practitioners towards fertility preservation among cancer patients, followed by a final section about sociodemographic information, such as participants' age, gender, and workplace. To validate the study questionnaire, a pilot study was performed to test the reliability and acceptability of the study and to confirm that the participants were able to understand each question in the same manner. In addition, to test the duration of time required to answer the questionnaire. For this, ten healthcare practitioners, who were experienced in treating cancer patients in Makkah region, were randomly selected and kindly asked to answer the same questionnaire. Their answers were then checked to detect if any variations might arise from the translation of the questions. According to the results of the pilot study, there were no modifications or omission of unnecessary or repeated questions. Health practitioners who participated in the pilot study were excluded from the study subjects.

RETRACTED

### 2.1. Statistical Analysis

Data entry and statistical analysis were done using the Statistical Package for Social Sciences software version 20.0 (SPSS Inc. Chicago, Illinois, USA). Mean and standard deviation were used to describe numerical data, and the percentage was used for categorical data. Frequencies of correct knowledge answers and various attitudes and practices were described. The Chi-square (*χ*^2^) test and Student's *t*-test were used for categorical data and continuous variables as appropriate. Results with a *P*value of <0.05 were considered statistically significant.

## 3. Results

One hundred healthcare practitioners who work with cancer patients in Makkah region agreed to participate in this study. The participants' age ranged from 25 to 65 years. The targeted population included both male and female practitioners (51% and 49%), respectively. Most of the study participants (75%) are working in Jeddah city, while 24% and 1% are working in Makkah and Taif city, respectively (Table 1).

As shown in Table 1, the demographic findings show a variety of cancer subspecialties among the study respondents of which, 30% were sub-specialized in gynecological cancer, followed by 24% in hematological cancer and other specialties.

Figure 1 shows the distribution of health practitioners according to their specialties. It appears that nurses were the most participating group (23%), followed by gynecologists (18%), surgeons (9%), medical oncologists (8%), and hematologists (8%). The results also show that other minor specialties accounted for less than 7% of total respondents. For example, radiation oncologists, anesthesiologists, fertility specialists, laboratory technicians and specialists, ophthalmologists, dermatologists, IVF consultants, clinical pharmacists, medical consultants, preventive medicine specialists, critical care doctors, pharmacists, and gastrologists.

Figure 2 illustrates the knowledge level of health practitioners regarding fertility preservation of cancer patients. The study reveals that 90% of the respondents need to raise their knowledge about fertility preservation in comparison to 10% who declared that they are knowledgeable. In addition, 51% of the participated health practitioners confirmed that they might be aware of fertility preservation, but they need to be knowledgeable about it. In contrast, 35% of respondents declared that they are knowledgeable or had adequate knowledge regarding fertility preservation. Among hundred participants, 14% declared that they do not know about fertility preservation. There was no significant association between health practitioners' knowledge and gender, age, workplace, and cancer subspecialty (all *P*values >0.05).

RETRACTED

With regard to fertility preservation procedures and options, data presented in Figure 3 reflect that most of the study participants (*n* = 87) were familiar with sperm freezing. The second, most commonly known option by health practitioners was egg freezing (*n* = 72). On the other hand, embryo, ovarian, or testicular tissue freezing, and GnRH-agonists pretreatment were the least fertility preservation options known to study respondents, (*n* = 39, 38, and 26, respectively).

Figure 4 displays the participants' attitudes regarding the most concerned gender about fertility preservation. Most health practitioners (*n* = 59) reported that both male and female populations considered fertility preservation options before cancer treatment. Among hundred participants, 26 health practitioners would consider women patients for fertility preservation, compared to 15 respondents who considered men patients to be the most concerned.

With regard to health practitioners' attitude in fertility preservation discussion, as demonstrated in Table 2 it appears that 66% of them agreed that fertility preservation was a high priority to be discussed with newly diagnosed cancer patients. In addition, 58% of study participants declared that they feel comfortable discussing fertility preservation with their patients. In contrast, few respondents disagreed with both statements (15% and 21%), respectively.

The study survey also included some questions about the success rates of fertility preservation and whether treating primary cancer is more important than fertility preservation. Around 54% of health practitioners agreed that treating cancer had a higher priority than fertility preservation. On the other hand, 21% disagreed with this statement. Nonetheless, the percentages of agreeing (36%) and disagreeing (41%) participants with the statement that fertility preservation is not a viable procedure for cancer patients due to its low success rates were nearly similar (Table 2).

The factors that influenced health practitioners' attitudes towards fertility preservation discussion with cancer patients are summarized in Table 3. It appears that more than 90% of health practitioners would discuss fertility preservation unless their cancer patient has a poor prognosis and/or cannot afford the expenses of fertility preservation. Other health practitioners declared further reasons that could affect their decision in discussing fertility preservation with their patients such as lack of fertility services in the patients' area (85%), the patient being too ill to delay treatment to pursue fertility preservation (85%), the patient is being diagnosed with hormonal sensitive malignancy (84%), or the patient already had a child or children (78%). On the other hand, the factors related to patients such as the inability to afford fertility preservation procedures or poor prognosis were among the least chosen reasons by study respondents that may affect their potential discussion with cancer patients (Table 3). There were significant associations between health practitioners' attitudes in discussing fertility preservation with their cancer patients and the influenced discussion factors (all *P*values <0.05).

RETRACTED

Figure 5 displays participants' attitudes towards fertility preservation practice guidelines. It appeared that among one hundred participants, 97% agreed with the need for fertility preservation practice guidelines (*P* < 0.001) compared to only 3% of participants who disagreed with the importance of creating fertility preservation practice guidelines (Figure 5).

Regarding fertility preservation referral, as illustrated in Figure 6 it appears that the majority of health practitioners (*n* = 69) (*P* < 0.01) are aware of a special clinic for fertility preservation or a specialist who will accept their referral compared to 31 individuals, who agreed that they are not aware of a particular clinic nor a specialist. Even though most of the respondents were aware, 46 did not refer any patient to fertility preservation (*P* < 0.05). On the other side, about 22 health practitioners declared that they referred up to 5 patients to fertility preservation. Furthermore, 32 confirmed that they referred more than five patients in the last five years (Figure 6). Independent sample *t*-tests and *χ2*-tests were also used to detect the association between participants' attitudes towards fertility preservation practice guidelines and their referral practice. There were significant relationships (all *P*values <0.05).

With regard to the most important factor for referring patients to fertility preservation, it appeared that many health practitioners (*n* = 25) consider the type of cancer, and (*n* = 22) select patient prognosis as the second most factor affecting their decision in referring the cancer patients. The cost and the patient's desire were among the most important factors for cancer patient referral, (*n* = 20 and 18), respectively. The bar chart also showed other less important factors such as the logistic issues, gender, time, and patient's marital status (Figure 7).

RETRACTED

In terms of participants' desire to have a free fertility preservation service for cancer patients provided by the Saudi Ministry of Health, it showed that most of the study participants (92%) agreed with the statement compared to 8% who disagreed with this notion (Figure 8).

## 4. Discussion

This study was conducted to assess the level of knowledge, attitude, and practice of health practitioners towards fertility preservation in cancer patients in Makkah region. The study indicates several significant findings. Firstly, the insufficient knowledge of health practitioners regarding fertility preservation could be mainly due to the lack of fertility preservation topics in medical education. Moreover, the national and private health care system in Saudi Arabia has focused only limited attention on fertility preservation. This highlighted the need to increase the knowledge regarding fertility preservation. The current finding was similar to the previous studies, which reported a lack of fertility preservation knowledge among health practitioners in France and Hong Kong.

Secondly, fertility preservation options such as sperm and oocyte cryopreservation appeared to be the most commonly known procedures among health practitioners. This is because these two options are the most recommended options by ASCO and the mostly used by doctors worldwide. For males, sperm cryopreservation is an effective and simple technique, which requires the production of a semen sample at any time before commencing the cancer treatment [7, 8]. However, in the female population, fertility preservation is more complex, costly, and time-consuming than in men. Oocyte or embryo freezing was more popular than ovarian tissue freezing among health practitioners. These findings were consistent with a previous study in Hong Kong, which found that the majority of health practitioners were familiar with sperm and oocyte freezing [8].

Thirdly, the current study showed that both females and males would be considered for fertility preservation. This highlights the fact that both genders are interested in reproduction and childbearing. This finding was in contrast to a previous study by Tschudin and Bitzer (2009), who reported that women were more interested in fertility preservation than men [31, 32].

Fourthly, most participating health practitioners declared that they are very likely to discuss fertility preservation with their cancer patients. However, many factors may significantly affect their attitude towards fertility preservation discussion such as poor patient prognosis or that the patient cannot afford the expenses of fertility preservation. These findings were in agreement with previous studies, which reported that the poor patient prognosis and the cost were among the factors that affected the health practitioners' attitudes to discuss fertility preservation with cancer patients [7, 8]. Moreover, the current study illustrates a low referring rate to fertility preservation. The reasons behind this could be related to the cancer type, patient prognosis, the cost, and the lack of fertility preservation centers in the patient area. Similar findings were also reported in a previous study conducted in Lebanon, where the clinicians had no choice but to not refer patients for fertility preservation due to the absence of well-developed fertility preservation centers [9].

RETRACTED

Furthermore, the majority of study participants agreed that fertility preservation and referring patients to such services should be associated with clear practice guidelines. This attitude can be explained by the lack of fertility preservation topics in general medical education and thus the need to increase the professional practical knowledge of fertility preservation. This result was consistent with a previous study in Hong Kong, which demonstrated a positive attitude and a great desire of health practitioners to establish fertility preservation practice guidelines [8].

In addition, most health practitioners in Makkah region agreed on the need for public fertility preservation services for cancer patients provided by the Saudi Ministry of Health. The cost of fertility preservation for a cancer patient plays an important role in the health practitioner's decision to discuss and refer the patient. In Saudi Arabia, the cryopreservation of sperms, oocytes, embryos, and other fertility preservation options are only available at private hospitals and a limited number of patients can afford it. Therefore, the Saudi Ministry of Health should consider providing these services to public or selected cancer patients. Clinicians in Hong Kong also agreed that patients have difficulties in paying for fertility preservation and suggested providing free clinics or centers for fertility preservation [8].

## 5. Conclusions

To our knowledge, this is the first study that assesses the knowledge, attitudes, and awareness of healthcare practitioners towards fertility preservation in cancer patients in Saudi Arabia, particularly in the Makkah region. As a result, healthcare practitioners' knowledge remains insufficient. Hence, further efforts are required to be conducted to ensure that the practitioners are discussing fertility preservation, its available options, and patients' referral to fertility preservation clinics before cancer treatments. This includes education, training programs, and increasing awareness campaigns regarding fertility preservation. Additionally, the establishment of well-developed fertility preservation services, referrals centers, and practice guidelines are recommended. Moreover, fertility preservation services should be provided as a free service to patients suffering from cancer. Such services should be funded by the Saudi Ministry of Health. Further studies in terms of cancer treatments risks and fertility preservation rights in Saudi Arabia are recommended [33].

RETRACTED

## Figures and Tables

**Figure 1:** Health practitioners' distribution according to their specialties. The pie chart shows that Nurses' health practitioners were the most participating health practitioners in this cross-sectional survey, followed by health practitioners who work as gynecologists, surgeons, medical oncologists, and hematologists.

**Figure 2:** Health practitioners' distribution according to their knowledge about fertility preservation. The bar chart shows that 90% need to raise their knowledge about fertility preservation, and 51% are aware of fertility preservation but they need to be knowledgeable about it.

**Figure 3:** Health practitioners' distribution according to their knowledge about fertility preservation available options. The bar chart shows that 87% of study participants were familiar with sperm freezing. The second, most commonly known option by health practitioners was egg freezing. On the other hand, embryo, ovarian, or testicular tissue freezing, and GnRH-agonists pretreatment were the least fertility preservation options known to study respondents.

**Figure 4:** Health practitioners' attitudes regarding patients most concerned gender about fertility preservation. The pie chart shows that 59% of study respondents reported that both males and females are equally concerned about fertility preservation options before cancer treatment, while 26% and 15% of study participants would consider women and men patients, respectively, for fertility preservation.

**Figure 5:** Health practitioners' attitude towards fertility preservation practice guidelines. The pie chart showed that 97% (*P* < 0.001) of the participants agreed with the need for fertility preservation practice guidelines compared to only 3% of participants who disagreed with the importance of fertility preservation practice guidelines.

**Figure 6:** Health practitioners' distribution according to their practice towards fertility preservation among cancer patients. The bar chart shows that 69% of participants are aware of a special clinic for fertility preservation or a specialist who will accept their referral (*P* < 0.01)*. E*ven though most of the respondents were aware, 46% did not refer any patient to fertility preservation during his/her last five years (*P* < 0.05).

RETRACTED

**Figure 7:** The most important factors in terms of patients' referrals according to the study participants. The bar chart shows that 25% and 22% considered the type of cancer and patient prognosis as the first and second most factors affecting their decision in referring the cancer patients, respectively. The cost and the patient's desire were also among the most important factors for a cancer patient's referral, while the logistic issues, gender, time, and patient's marital status were less important factors.

**Figure 8:** Health practitioners' opinions regarding fertility preservation service. It showed that 92% of the study participants agreed with the statement, compared to 8% who disagreed with this notion.

**Table 1:** Distribution of study participants according to their demographic characteristics.

Characteristics	Participants number	
	No.	%
*Gender*		
Female	49	49
Male	51	51
*Age*		
25–35	38	38
36–45	31	31
46–55	15	15
Over 55	16	16
*Workplace*		
Makkah	24	24
Jeddah	75	75
Taif	1	1
*Cancer subspecialty*		
Gynecological	30	30
Hematological	24	24
Breast	16	16
Pediatric	13	13
Lung	4	4
CNS	3	3
Urological	3	3
Gastrointestinal	3	3
Sarcomas/soft tissue	3	3
Head and neck	1	1

**Table 2:** Health practitioners' attitude in discussing fertility preservation with their cancer patients.

Health practitioners' attitude	Agreement no. (%)	Neither no. (%)	Disagreement no. (%)
Fertility preservation is a high priority for me to discuss with newly diagnosed cancer patients	66 (66%) (*P* < 0.05)	19 (19%)	15 (15%)
I feel comfortable discussing fertility preservation with my patients	58 (58%) (*P* < 0.05)	21 (21%)	21 (21%)
Treating the primary cancer is more important than fertility preservation	54 (54%) (*P* < 0.05)	25 (25%)	21 (21%)
The success rates of fertility preservation are not as yet good enough to make it a viable option	35 (36%)	24 (24%)	41 (41%)

**Table 3:** Factors influence health practitioner's discussion of fertility preservation with their cancer patients.

Factors	Agreement	Disagreement No. (%)
	No. (%)	
The patient cannot afford fertility preservation	92 (92%) (*P* < 0.001)	8 (8%)
The patient has a poor prognosis	91 (91%) (*P* < 0.001)	9 (9%)
Lack of fertility services in the area	85 (85%) (*P* < 0.001)	15 (15%)
The patient is too ill to delay treatment to pursue fertility preservation	85 (85%) (*P* < 0.001)	15 (15%)
The patient has a hormonally sensitive malignancy	84 (84%) (*P* < 0.001)	16 (16%)
The patient already has a child or children	78 (78%) (*P* < 0.001)	22 (22%)
The patient does not want to discuss fertility preservation	77 (77%) (*P* < 0.001)	23 (23%)
Constraints on my time	72 (72%) (*P* < 0.001)	28 (28%)
Someone else within my practice discusses fertility preservation with my patients	70 (70%) (*P* < 0.001)	30 (30%)
My limited knowledge of fertility preservation options	69 (69%) (*P* < 0.001)	31 (31%)
The patient is single	57 (57%) (*P* < 0.001)	43 (43%)

RETRACTED

## Data Availability

The datasets used and/or analyzed during the current study are available from the corresponding author upon reasonable request.

## Abbreviations

ASCO: American society of clinical oncology
ART: Assisted reproduction technologies
°C: Celsius
CNS: Central nervous systems
DNA: Deoxyribonucleic acid
F.P: Fertility preservation
GCO: Global cancer observatory
GnRH: Gonadotropin-releasing hormone
IVF: In vitro fertilization
ICSI: Intracytoplasmic sperm injection
IUI: Intrauterine insemination
MOH: Ministry of health
NHL: Non-hodgkin lymphoma
WHO: World health organization.
